# Novel Crow Swarm Optimization Algorithm and Selection Approach for Optimal Deep Learning COVID-19 Diagnostic Model

**DOI:** 10.1155/2022/1307944

**Published:** 2022-08-13

**Authors:** Mazin Abed Mohammed, Belal Al-Khateeb, Mohammed Yousif, Salama A. Mostafa, Seifedine Kadry, Karrar Hameed Abdulkareem, Begonya Garcia-Zapirain

**Affiliations:** ^1^College of Computer Science and Information Technology, University of Anbar, Ramadi 31001, Anbar, Iraq; ^2^Directorate of Regions and Governorates Affairs, Ministry of Youth & Sport, Ramadi 31065, Anbar, Iraq; ^3^Faculty of Computer Science and Information Technology, Universiti Tun Hussein Onn Malaysia, Johor 86400, Malaysia; ^4^Department of Applied Data Science, Noroff University College, Kristiansand 4608, Norway; ^5^College of Agriculture, Al-Muthanna University, Samawah 66001, Iraq; ^6^College of Engineering, University of Warith Al-Anbiyaa, Karbala, Iraq; ^7^eVIDA Laboratory, University of Deusto, Avda/Universidades 24, Bilbao 48007, Spain

## Abstract

Due to the COVID-19 pandemic, computerized COVID-19 diagnosis studies are proliferating. The diversity of COVID-19 models raises the questions of which COVID-19 diagnostic model should be selected and which decision-makers of healthcare organizations should consider performance criteria. Because of this, a selection scheme is necessary to address all the above issues. This study proposes an integrated method for selecting the optimal deep learning model based on a novel crow swarm optimization algorithm for COVID-19 diagnosis. The crow swarm optimization is employed to find an optimal set of coefficients using a designed fitness function for evaluating the performance of the deep learning models. The crow swarm optimization is modified to obtain a good selected coefficient distribution by considering the best average fitness. We have utilized two datasets: the first dataset includes 746 computed tomography images, 349 of them are of confirmed COVID-19 cases and the other 397 are of healthy individuals, and the second dataset are composed of unimproved computed tomography images of the lung for 632 positive cases of COVID-19 with 15 trained and pretrained deep learning models with nine evaluation metrics are used to evaluate the developed methodology. Among the pretrained CNN and deep models using the first dataset, ResNet50 has an accuracy of 91.46% and a F1-score of 90.49%. For the first dataset, the ResNet50 algorithm is the optimal deep learning model selected as the ideal identification approach for COVID-19 with the closeness overall fitness value of 5715.988 for COVID-19 computed tomography lung images case considered differential advancement. In contrast, the VGG16 algorithm is the optimal deep learning model is selected as the ideal identification approach for COVID-19 with the closeness overall fitness value of 5758.791 for the second dataset. Overall, InceptionV3 had the lowest performance for both datasets. The proposed evaluation methodology is a helpful tool to assist healthcare managers in selecting and evaluating the optimal COVID-19 diagnosis models based on deep learning.

## 1. Introduction

In December 2019, a new coronavirus called (COVID-19) was appeared in China, particularly in Wuhan. The COVID-19 spread worldwide caused disastrous effects and lead to death [1]. COVID-19 pandemic gets great attention from global and health institutions as it has no cure yet [2]. COVID-19 consists of RNA-type with positive-oriented single-stranded, making finding the treatment challenging because of the mutating characteristics [3]. Scientists and researchers have created a hard effort worldwide to discover an effective treatment for COVID-19. According to the global statistical data, China, the USA, Brazil, Italy, Spain, Iran, the UK, and many other countries have lost thousands of persons due to the COVID-19 [4]. The coronavirus family has different types, and they can infect animals. This issue includes COVID-19, which can be seen in bats, poultry, rodent, cat, dog, pigs, and humans. The common COVID-19 symptoms are fever, dry cough, headache, sore throat, runny nose, and muscle pains. Infected people with COVID-19 who have weak immune systems are the potential to die. COVID-19 can infect healthy people through physical contact such as breath, mucous, and hand contact with infected people [5].

Different diagnosis biomarkers have been used in the detection of COVID-19, such as blood test samples, X-ray, breathing recordings, ultrasound images, nuclear medicine imaging, and CT images [1]. For the regions that were early attacked by the COVID-19 pandemic, RT-PCR can be an inappropriate examination. As reported in [6], some lab COVID-19 examinations are deficient in sensitivity with 71%, which is based on many factors, including quality control and sample preparation. Other radiology examinations, including thoracic CT and lung X-ray, positively help the medical practitioners in COVID-19 diagnosis [7]. Many cases in China diagnosed with COVID-19 have shown some abnormalities in the CT scans [8]. People who are suspected of COVID-19 infection with no apparent symptoms ask to quarantine to make more COVID-19 examinations. In the context of examination sensitivity, people who are suspected of COVID-19 infection must make a nucleic acid test several times to confirm the COVID-19. The results of imaging examinations are essential to combat the COVID-19 slowdown it is speared. Radiological imaging is the most rapid, accurate examination for COVID-19 diagnosis. By using computed tomography (CT) imaging, to detect any abnormalities, most of the cases share the same characteristics, including a rounded morphology and a peripheral distribution. Also, pulmonary consolidation appears in the advanced stage, and ground-glass opacities appear in the early stage [7]. CT imaging examination can assist radiologists and doctors in diagnosing COVID-19 early. However, sometimes radiologists and doctors find it difficult to diagnose COVID-19 based on CT images as the viral cases of pneumonia look like other inflammatory diseases in the lung. Concerning imaging-based COVID-19 examination, particularly CT imaging, there are three diagnosis workflow stages: pre-scan preparation stage, acquisition of image stage, and final diagnosis of disease stage. In the first stage, the patient is prepared and instructed for bed examination based on a certain protocol. The CT images are scanned in the image acquisition stage, and the patient is requested to hold their breath during the scan process, which covers the area of the upper lung through the lung base. The radiologists set the proper measurements of the area that would be covered in the scan based on the body shape of the patient. CT images are generated from the obtained raw data. Then they are processed via picture archiving and communication system (PACS) for diagnosis. Artificial intelligence (AI) can positively be incorporated with medical imaging to help in the COVID-19 diagnosis and combat the disease [9]. In contrast to the classical imaging tool procedures, which mainly depend on technicians and radiologists, imaging tools incorporated with AI are less human dependent and more accurate, safer, and efficient. The modern AI-driven system for COVID-19 diagnosis has a dedicated imaging platform, segmentation of the infected areas, and various diagnosis and evaluation tools. Furthermore, AI technology is embedded successfully in various commercial systems to fight COVID-19 and use this advanced technology. In February 2020, the first virtual seminar on COVID-19 was organized by the Medical Imaging Computing Seminar (MICS), an alliance of medical imaging scholars and start-up companies in China. Thousands of interested people attended the seminar. Those examples indicate how strong the public interest regarding the utilization of the AI in the imaging field for medical purposes to fight COVID-19.

Optimization methods and AI models have a great capability to combat COVID-19 by obtaining more accurate and reliable diagnoses in a short and optimized time efficiently. In recent times, many AI-based computer-assisted systems have been used in various medical institutions and hospitals to diagnose COVID-19 automatically rather than the traditional manual method of data analysis. Although many AI methods are utilized in automated COVID-19 systems, it is a big challenge for medical institutions and hospitals to select the best method that meets their needs and produces reliable and accurate results [10]. However, there is no AI-based model better than others [11]. The challenge becomes more prominent when the hospitals and healthcare managers need to evaluate the AI-based model with various metrics. Furthermore, many deep learning detection models are designed for COVID-19 diagnosis. Healthcare managers face difficulty selecting the appropriate method, evaluating it with different metrics, and validating the medical solutions. A wrong solution has devastating effects that might lead to losing a patient's life, financial crisis, and legal accountability. For instance, if the AI-based model obtains the wrong result and shows a positive COVID-19 for the noninfected healthy person, the person will receive unnecessary treatment with side effects. In contrast, if the AI-based model obtains the wrong result and shows a negative COVID-19 for the infected person, the patient will not receive the correct cure, and their health condition might be worsening. In addition, the patient infects the other noninfected people. Both examples have severe consequences for the hospitals and healthcare institutions concerning credibility and reputation. Therefore, selecting a diagnostic AI model that produces free errors, reliable, and non-costly solutions is therefore essential. Moreover, making an evaluation is not a trivial task, especially when various measurements are involved. Group reliability and time complexity are two popular criteria that must be considered to evaluate deep learning models of COVID-19 diagnosis. Concerning group reliability, many measures can belong to group reliability, including *F*1-score, precision, average accuracy, recall, error rate, true negative (TN), false negative (FN), true positive (TP), and false positive (FP) [12]. According to [13], the accuracy criterion has been used to evaluate various deep learning models, such as studies in [14]. The evaluation of the deep learning model for COVID-19 diagnosis is not only restricted to accuracy criteria. There are multiobjective/criteria that must be considered in the evaluation when selecting the optimal model.

This study proposes an integrated evaluation methodology for different COVID-19 diagnosis models based on deep learning. The method motivates the authors to develop integrated deep learning classifiers under one framework and involves the most common performance evaluation criteria of COVID-19 diagnosis models based on deep learning. The proposed evaluation methodology is a helpful tool to assist healthcare managers in selecting and evaluating the optimal COVID-19 diagnosis models based on deep learning. The main contributions of this study can be summarized as follows:

- An integrated method is proposed for selecting the optimal deep learning model based on the novel crow swarm optimization (CSO) algorithm for COVID-19 diagnosis.
- The crow swarm optimization (CSO) is employed to find an optimal set of coefficients using a designed fitness function for evaluating the performance of the deep learning model. The CSO is modified to obtain a good distribution of selected coefficients by considering the best average fitness.
- In order to show its performance, CSO is benchmarked with some well-known swarm optimization algorithms, those are Grey Wolf Optimization (GWO), Harris Hawks Optimization (HHO), Salp Swarm Algorithm (SSA), and Whale Optimization Algorithm (WOA).
- We have utilized two datasets: the first one includes 746 CT images, 349 of which are of confirmed COVID-19 cases and the other 397 are of healthy individuals; and the second dataset composed of unimproved CT images of the lung for 632 positive cases of COVID-19 with 15 trained and pretrained deep learning models with nine evaluation metrics used to evaluate the proposed methodology.
- Deep convolutional CNN feature representation is applied to extract highly representative features via successful descriptors of deep CNN. Our proposed method can distinguish between the infected region of COVID-19 and the noninfected region in the lung CT scan and X-ray images, which improves the accuracy compared to other existing methods. To the best of the authors' knowledge, this work is the first inclusive study, including 15 deep learning classifiers.
- The devolved method minimizes the classification time significantly while yielding higher accuracy. This is a great benefit when developing an automatic real-time medical system.

The rest of this article is organized as follows: Section 2 presents the related works of the COVID-19 diagnostic systems highlighting the initial associated studies. The developed selection methodology for COVID-19 diagnostic models is proposed in Section 3. The experimental result of the proposed COVID-19 diagnostic selection methodology based on the CSO algorithm is provided in Section 4, with the study limitation and future work. Finally, conclusions have been provided in Section 5.

## 2. Related Works

COVID-19 is caused by severe acute respiratory syndrome corona virus 2 (SARS-CoV-2). It first appeared in Wuhan city in China in late 2019 [15]. As a result of the COVID-19 pandemic, scientists and researchers in the medical and healthcare community are dedicating efforts to finding a solution to fight COVID-19 and control the spreading rate [16]. Several COVID-19 related studies are proposed to assess pneumonia caused by COVID-19 and the degree of COVID-19 infection to make the appropriate decision regarding the treatment plan and select the appropriate medication and required doses. Hospitals and medical centers widely used noninvasive image methods such as X-ray and lung CT scans to detect COVID-19 pneumonia severity. The result of CT images is more precise compared to X-rays. Therefore, this work is limited to the CT scan imaging (CTSI) examination only. Moreover, the CTSI provides more accurate results than reverse transcription-polymerase chain reaction (RT-PCR). There are massive studies presented recently that proposed detection and prediction methods for COVID-19 diagnosis [17]. In [4], a deep review of the prediction and detection methods for COVID-19 is presented. The review also includes laboratory-level detection methods such as RT-PCR and CTSI physical assessment reported by skilled radiologists. The automatic detection method produces a rapid and accurate solution with no need for a hard-human labor effort.

In [18], a deep learning-based method, namely VIDX-Net, is developed for COVID-19 diagnosis using chest X-ray images. Comparative study of various deep learning classifiers including DenseNet and other models is discussed in detail for esNetV2, MobileNetV2, and InceptionV3 with proposed images dataset provided for public use. It consists of 50 X-ray images, half of them belong to the health cases while the other half belong to the COVID-19-infected cases [19]. The result in [20] shows DenseNet201 and VGG19 classifiers perform better than other classifiers with an accuracy of up to 90.00%. A COVID-19 diagnostic model based on machine learning is proposed in [21]. The proposed model used 150 CT images divided into different groups, including 16, 32, 48, and 64. The study also uses various handcrafted features, including discrete wavelet transform (DWT), grey level co-occurrence matrix (GLCM), grey level size zone matrix (GLSZM), local directional pattern (LDP), and grey level run length matrix (GLRLM). A support vector machine (SVM) classifier is employed in the study of [21]. SVM was inserted the extracted features based on different cross-validations (2-fold, 5-fold, and 10-fold). The extractor of GLSZM features achieved a higher accuracy, which equals 98.77% of 10-fold cross-validation. A deep learning-based COVID-Net method using lung X-ray images for the detection of COVID-19 is presented in [22]. The proposed method's structure combined one-one convolutions, the residual modules, and depthwise convolution to allow a deeper architecture and overcome the gradient vanishing problem. The proposed method used a combination of COVID-19 lung X-ray dataset obtained from [23] with different classification groups, including normal class, viral infection (non-COVID-19), COVID-19, and bacterial infection. The accuracy of the method reached up to 83.5%.

An automatic COVID-19 diagnostic approach based on deep learning and transfer learning strategy is proposed in [24]. The proposed approach's structure combines a convolutional neural network (CNN) and a modified AlexNet [25] with the feasibility of transfer learning. The CNN architecture comprises one convolutional layer, batch normalization with 16 filters, two fully connected layers, and a rectified linear unit (ReLU). The proposed combination approach can obtain accuracy up to 94.00%. An investigation of interpretability of deep learning-based models and uncertainty of COVID-19 diagnostic detection using X-ray images is conducted in [26]. Bayesian convolutional neural network (BCNN) and drop weight mechanism are used to estimate deep learning uncertainty. This combination can increase the clinical practice trust by achieving consistent results. The proposed method to assess the correlation between uncertainty and accuracy uses 70 chest X-ray images of COVID-19 cases which are obtained from public datasets of [23]. The dataset is prepared, and the size of all images is adjusted to 512 pixels. A real-time data augmentation strategy and transfer learning strategy are used to deal with the limitation of the dataset size. The proposed approach is achieved accuracy up to 94.00% when applied VGG16 deep learning method. A transfer learning strategy of a 10-fold cross is combined with a VGG16 architecture in [27]. The proposed model trained using the dataset obtained from [19]. The size of all images is adjusted to 224 pixels. The real-time data augmentation strategy is used to overcome the limitation of the dataset size. The proposed method obtained 96.1% and 99.70% in accuracy and area under the curve (AUC), respectively. A new architecture of fine-tuned and pretrained ResNet50 for COVID-19 is proposed in [28]. The proposed model involved various data augmentation strategies, including random rotation and vertical flip, to enhance the training model generalization. The proposed model yielded accuracy up to 96.23% on a multiple class, including COVID-19 infection, normal, viral infection, and bacterial infection dataset.

For controlling the spread, an initial diagnosis of alleged COVID-19 cases and screenings must be carried out daily as shown in related COVID-19 diagnosis reviews or literature. For a rapid and accurate diagnosis of COVID-19, extraction of radiological features using AI and ML has proven the principle's efficacy as observed in the outcomes. In carrying out clinical diagnoses, the use of X-ray and computed tomography (CT) images essentially provide useful information. This necessitates, therefore, that doctors have an automatic CT image diagnosis system developed to help them in COVID-19 diagnosis. According to [29], a two-stage data enhancement method must be used in classifying the images of coronavirus and five other situations. Due to unbalanced and deficient image numbers in the dataset, the initial phase applied the use of a shallow image augmentation method. Feature extraction using handcrafted approaches come in more useful and convenient in analyzing these images because of the insufficiency of the newly created dataset in deep architecture training. Furthermore, in the study, the next data enhancement phase utilizes an algorithm called the synthetic minority over-sampling method. Conclusively, a stacked autoencoder and principal component evaluation technique is applied to resize the feature vector *y* by removing interlinked or associated features present in the feature vector. As in the obtained results, it is observed that COVID-19 diagnosis can be performed effectively and quickly due to the proposed model's performance leveraging capability.

COVID-19 and other atypical and viral (non-COVID-19) respiratory diseases appear indistinguishable in comparison. A clinical computer-aided diagnosis (CAD) system in the study by [30] applies automatic discrimination of COVID-19 from non-COVID-19 pneumonia patients using CT features. A total of 612 recruitment containing 306 COVID-19 and 306 non-COVID-19 cases were made. From the CT images, extraction of 20 radiological features was performed, and these features were used for the pattern, location, and lesions' distribution evaluations of patients in groups. To evaluate the CAD system with best performance and classification of COVID-19 and non-COVID-19 cases, support vector machines, naïve Bayes, decision tree, k-nearest neighbor, and ensemble are five classifiers trained using all the significant CT features. These significant COVID-19 groups are air bronchogram, cavity, consolidation, crazy-paving, and ground-glass opacity (GGO), involvement distribution pattern and location, lesion numbers, lymphadenopathy, nodule, pleural effusion, and thickening, reticular, and thickening of the bronchial wall. On implementation using an ensemble COVIDiag classifier, an accuracy of 91.94%, a sensitivity of 0.965, and specificity of 93.54% were observed in the proposed CAD system. A COVIDiag model, as suggested by this study using CT radiological routine features, provided results that are encouraging in COVID-19 diagnosis. The study claims that radiologists can consider using this tool as support in making better and accurate COVID-19 diagnoses in this present pandemic. [31] came up with a diagnosis framework called CovidCTNet in an attempt to better CT imaging detection accuracy. CovidCTNet comprises a set of deep learning algorithms that accurately distinguish COVID-19 from any community-acquired pneumonia (CAP) or other respiratory ailments. CovidCTNet obtained an accuracy of 95% in CT imaging detection as to 70% obtained from radiologists. Independent of the CT imaging device, CovidCTNet is embedded with the ability to work with heterogeneous and small sample size data. [31] made available in open source the model metrics and all algorithms in detail to more trustworthy the detecting capacity of COVID-19 globally and support radiologists and doctors during the screening procedures. While CovidCTNet's sharing helps to preserves data ownership and user confidentiality, it further facilitates rapid improvement and service optimization by developers. Another study by [32] concentrated on applying different deep learning methods to distinguish between COVID-19 and non-COVID-19 CT scan images. As a result, a CTnet-10 model with an accuracy of 82.1% was self-developed and designed. Furthermore, other models including DenseNet169, InceptionV3, ResNet-50, and VGG19 were tested. VGG19 came up with a superior accuracy of 94.52% among the trialed deep learning techniques from the results. For rapid and effective screening for COVID-19 diagnosis, automated COVID-19 diagnosis from CT scan images can prove a useful method to doctors.

In the work of [33], 1065 CT pictures of previously diagnosed patients with common viral pneumonia and pathogen-confirmed COVID-19 cases were obtained. The inception transfer learning model was modified to develop the algorithm and further carried out the internal and external validation. An accuracy of 89.5%, specificity of 88.0%, and sensitivity of 87.0% were obtained for the internal validation. In the external validation, the accuracy, specificity, and sensitivity showed 79.3%, 83.0%, and 67.0%, respectively. More so, the algorithm with 85.2% accuracy detected 46 out of 54 COVID-19 images as COVID-19 positive, with the first two nucleic acid test outcomes were negative. Similarly, the work of [34] obtained CT images of 262 persons for COVID-19, 100 persons for bacterial pneumonia, 219 persons for common viral pneumonia, and 78 persons for healthy control. They combined the newly developed ResNet50 backbone and SE blocks for image analysis to come up with a model that can effectively detect and obtain the indefinite or abstruse differences in CT images. This model produced accuracy, AUC, recall, precision, and *F*1-score of 94%, 0.96, 0.94, 0.95, and 0.94, respectively, which shows superior performance compared to the generally utilized basic models.

Based on this review for the recent COVID-19 diagnosis deep learning or machine learning methods using CT or X-ray image classification, several open research issues need further studies. The first issue is that there is no standard and certified CT or X-ray image dataset with the quality and quantity of the images to produce reliable results. The second issue is there is no deep learning or machine learning model that can yield the best results. Each of the proposed models might produce acceptable to high results in certain circumstances. The third issue is determining the main constrain of the existing models that affect the performance and the diagnosis quality. Most AI-based COVID-19 are not available for public use to the best of the authors' knowledge, which does not allow the researchers to use them in the research. However, some other researchers attempt to make COVID-19 radiography imaging and COVID-19 diagnosis model based on AI and deep learning that are accessible for the research community. The COVID-19 chest CT and X-ray dataset are publicly available now. Evaluation of the deep learning-based models with the group reliability and the time complexity of time is a necessity to assess their quality. ML-based models that used radiography can produce more accurate and reliable results [35].

[36] propose a classification method of COVID-19 based on CT images. The method integrated CNN with transfer learning and sparrow search algorithm (SpaSA) for hyperparameter optimization. The transfer learning is used to initialize the CNN training cycle, and the SpaSA is used to select the best trained model. The method has achieved the best accuracy of 99.74%. Also, the study made by [37] focuses on identifying the state-of-the-art computational algorithms for diagnosing COVID-19. The study claims that CT images can provide the means for the early detection of COVID-19. Moreover, the computational algorithms' ability to detect COVID-19 is highly affected by detecting certain visual features in the CT images, such as the ground‐glass opacity (GGO) feature. The study concludes with the need for the initial training of the deep learning algorithms to overcome the unavailability of sufficient training samples. Another work by [38] propose a CNN model with depthwise separable dense and convolution block attention module. The convolutional block attention module is used to extract high-quality features that help to overcome the overfitting of the training model. The depthwise separable dense is used to reduce the dimensionality of the features and support lightweight prediction models. The model has been tested on a small sample of X-ray and CT images and is able to achieve an accuracy of 98.62% and 99.18, respectively. It is able to reduce training parameters and outperforms four similar models. The work of [39] attempts to evaluate the performance of four machine learning models, namely decision tree (DT), partial least squares discriminant analysis (PLS-DA), artificial neural network (ANN), and K-nearest neighbor algorithm (KNN), in COVID-19 diagnosis and severity. The used data for testing are laboratory tests results of patients (557 positives and 5,086 negatives COVID-19). The accuracy of the four tested models has exceeded 84%, and the ANN model achieves the best performance of 96% accuracy on average.

In the literature, numerous studies are presented that deal with radiography imaging for COVID-19 diagnosis. But no such study deals with evaluating the diagnostic system based on deep learning models to assist the healthcare managers in selecting the optimal COVID-19 diagnostic system. This work attempts to bridge the gap between the selections of COVID-19 diagnostic ML-based model and radiography imaging. This study proposed automatic COVID-19 detection deep learning-based models using chest CT images. This motivates the authors to employ 15 deep learning models, including MobileNets V2, VGG19, DarkNet, ResNet50, Xception, GoogleNet, ResNet34, SAE, CNNs, InceptionResNetV2, NASNet-Large, InceptionV3, LSTM, and DNN, to find the optimal accuracy using 746 chest CT images dataset. Also, in this study, we compute 9 evaluation measurements, including classification accuracy rate (CAR), predictive positive value (PPV), *F*1-score, false positive rate (FPR), mean squared error (MSE), precision, AUC (area under the curve), negative predictive values (NPV), recall, and ROC (receiver operating characteristics) curve. The crow swarm optimization (CSO) is employed in this study to find an optimal set of coefficients based on a designed fitness function for the evaluation the deep learning performance. CSO acts as a distribution strategy to ensure all the selected coefficients are distributed fairly by considering only the best available average fitness.

## 3. Methodology

Rapid and correct diagnosis of COVID-19 possible cases performs a vital role in quarantine and treatment systems. Exacting quick, exceptionally early diagnosis results of COVID-19 suspected cases plays a significant part in inconvenient isolation and treatment, which is also of extraordinary significance for patients' guesses, the control of this scourge, and the open well-being security. But right now, a huge number of suspected patients must experience chest CT checking. This process has caused a huge burden to proficient therapeutic staff. Their extreme deficiency is also a major challenge within the current circumstance; additionally, radiologists' visual weariness would increase the potential dangers of failure in diagnosing all the cases. Developing a computerized detection system based on CT lung scan images is valuable to counter the outbreak of COVID-19 or SARS-CoV-2. The previous studies like [40] show that with a considerable small simple of scanned CT lung scan images between 500 and 800, different types of DL algorithms are able to detect COVID-19 cases with high accuracy [41]. Subsequently, this research proposes an automatized deep learning-based COVID-19 detection system. The study aims to investigate the most optimal DL model for a more effective COVID-19 detection system in comparison to the latest DL computer-aided diagnosis methods. The proposed selection method for the best DL models is shown in Figure 1. Also, pseudocode for the selection approach for optimal deep learning COVID-19 diagnostic model using CSO approach is presented in Algorithm 1. The methodology section is divided into three main sections as follows:

### 3.1. Development Stage

#### 3.1.1. CT Lung Scan COVID-19 Dataset

In this study, we have utilized two datasets to validate our methods. The first dataset includes 746 CT images, 349 of them are confirmed COVID-19 cases and the other 397 are of healthy individuals [19]. The CT images and other references and resources are mainly taken from free and open access websites such as medRxiv and bioRxiv. The primary COVID-19 dataset collection of our work covered the period from January 19 to May 25 2020. The COVID-19 cases of the dataset comprise a full clinical depiction of the patients' conditions. A case of chest CT images for patients having COVID-19 is presented in Figure 2.

The second dataset is the NIfTI retroactive dataset composed of the lung's unimproved CT images for 632 positive cases of COVID-19. These images are obtained from a medical care center for people who show a reverse transcription-polymerase chain reaction (RT-PCR) to confirm the COVID-19 infections at the rapid spread of the corona pandemic. Patient severing with some symptoms of COVID-19 are caused by direct contact with an infected people or travel to countries affected by Corona. Initial CT examination of the suspected patients confirms the positive COVID-19 cased based on RT-PCR. A soft tissue rebuilding algorithm is used to examine the CT images with no need for vascular contraindication. At a subsequent time, all DICOM images are transformed into the format of NIfTI [42].

#### 3.1.2. Deep Learning Models

Recently, one of the tremendously expanding machine learning algorithms in medical imaging research is DL [43]. It has achieved significant diagnostic outcomes in different disease detection types, including cancers and brain, heart, and lung diseases [44]. The different image-based datasets such as ImageNet introduces millions of images as training and testing dataset [45]. For instance, in 2020 [46], DL models show dermatologist-level execution on classifying skin lesions. In 2018, the DL model of [47] produced exceptional outcomes for diagnosing breast cancer from image screening. However, in many cases, the most profound learning-based algorithms for infection determination require explaining the lesions, particularly for infection location in the CT volumes. There are several breakthroughs of DL neural network models that outperform human-level execution. Subsequently, in this study, 15 DL models are selected to investigate the best suitable model for COVID-19 diagnosis comprehensively. The models are convolution neural network (CNN), DarkNet, deep neural network (DNN), GoogleNet, InceptionResNetV2, InceptionV3, LSTM, MobileNetV2, NASNet-Large, ResNet34, ResNet50, Stacked autoencoder (SAE), VGG16, VGG19, and Xception. They are briefly described in Table 1 and explained in the following. Also, the parameters of the COVID-19 deep learning models have been listed in Table 2.

- Convolution Neural Network: The convolution neural network (CNN) is a multilayer neural network consisting of a set of fully connected layers and convolution layers. The convolution layers are the standard layers of the CNN. The CNN's basic concept includes perception, weights, and sampling (time or space), which backs to the early 60 s [48]. The CNN and the neural network, in general, have a local perception that efficiently detects the local feature of the data or object in an image. The CNN input parameters are usually fewer than the hidden layers, which makes it less data dependent.
- DarkNet: The DarkNet DL model is designed based on state-of-the-art Darknet-19 architecture. The Darknet-19 type is a classification model that has been made for the YOLO tool to perform real-time object detection. This system has an architecture designed for object detection [49].
- Deep Neural Network: The deep neural network (DNN) is a type of neural network that conducts intensive computation to its input because of nonlinear transformation in its hidden layers. Unlike the conventional neural network, the hidden layers encompass nonlinear functions for further analysis. The DNN has many hidden nodes compared with the conventional neural network. Subsequently, it takes a longer execution time and produces more accurate results [50].
- GoogleNet: The GoogleNet is a DL model that uses very few input parameters. It is tested on Places365 and ImageNet datasets for object detection and found to be efferent in terms of accuracy and execution time. The GoogleNet model network consists of 22 layers (three convolution layers, nine inception blocks, and the rest are fully connected layers) [51].
- InceptionResNetV2: The InceptionResNetV2 is a CNN model that includes numerous types of pooling and convolution layers. As in many other models, it contains fully connected layers before the output layer. The early InceptionResNet model has been recognized as one of the top CNN models based on different benchmark datasets such as the ImageNet dataset and JFT Google internal datasets [52]. The InceptionResNetV2 is known for its efficient execution to low-level operations and scalability to fit with a different type of application.
- Inceptionv3: The Inceptionv3 is the third generation of Google's Inception CNN that initially introduced a module for GoogleNet. It is tested in the ImageNet Recognition Challenge of visual object detection and image analysis. It is very popular in classifying visual objects for computer vision applications [53].
- LSTM: The LSTM is a type of recurrent neural network (RNN) proposed by Hochreiter and Schmidhuber to deal with sequences of data efficiently. It uses gates to regulate the input data before the learning and remembering process. However, the gates might filter out important data that affect the network's performance [53].
- MobileNetV2: The MobileNetV2 is the second version of the MobileNetV1 DL neural network included in the TensorFlow-Slim Image Classification, Collaboratory, and some other alternative libraries. It has lower complexity and model size compared with the MobileNetV1. Google proposes it for mobile phone visual recognition applications to perform object detection, classification, and semantic segmentation [53].
- NASNet-Large: The NASNet-Large is a CNN model that is trained to classify 1000 objects based on the ImageNet database that contains several millions of images [53]. It can transfer learning to classify objects of new untrained images. The network receives images of the 331-by-331 size and extracts features of objects such as a computer mouse, keyboard, pencil, animals, etc.
- ResNet34: The ResNet34 is an improved version of the residual neural network (ResNet) base model with 34 layers. The ResNet has a CNN architecture but with a shortcut mechanism between layers to speed up solving problems. The shortcut mechanism prevents alteration and reduces the complexity of the network. Moreover, the ResNet model has a bottleneck blocks mechanism to speed up the network's training process [53].
- ResNet50: The ResNet50 is another version of the ResNet with 50 layers. It differs from the ResNet34 by trending to perform deeper analysis to solve complex problems, and hence it has better object classification and recognition accuracy. However, in many cases, a deeper analysis degrades the accuracy of the network. As with many other CNN models, the ResNet50 is tested using the ImageNet dataset to recognize and classify objects and shows high-quality performance [53].
- Stacked autoencoder: The stacked autoencoder (SAE) is a multilayer DNN that entails input, hidden, and output layers. The number of neurons in the input layer and output layer are equal, and the hidden layer usually has lesser neurons than them. The SAE has an unsupervised learning algorithm that differs from other networks by a stacked autoencoder [54]. The stacked autoencoder performs a coding and decoding process in which the coding takes place for the data of the input and the hidden layers, while decoding takes place for the data of the hidden and the output layers. The SAE provides a feature fusion mechanism that enables it to deal with a small dimension of features.
- VGG16: The VGG16 is another type of CNN model (a variant of the main VGG model, including VGG11 and VGG19) that consists of 16 layers. Simonyan and Zisserman propose it for processing large-scale image recognition tasks. It differs from the AlexNet model by integrating multiple 3 × 3 kernel-sized filters instead of kernel-sized filters in the convolutional layers. It produces considerably high accuracy results than some other popular models but with the cost of longer training time. The VGG16 model achieves an accuracy of 92.7% when applied to the ImageNet challenges and scores a place in the top 5 CNN models [55].
- VGG19: The VGG19 is another variant of the main VGG model, which consists of 16 convolution layers, 5 MaxPool layers, 3 fully connected layers, and 1 SoftMax layer (i.e., 19 layers in total). The input to the VGG19 is an RGB image of a fixed size (224 ∗ 224) that is represented by a (224, 224, 3) matrix [56].
- Xception: The Xception is a recent CNN model that is inspired by the InceptionResNet [39]. The InceptionResNet, Inceptionv3, and later Xception are characterized by the addition of the Inception module, but its have different versions of various parameters [18]. The improvements of the Xception enable it to slightly outperform the older version when applied to the ImageNet dataset.

#### 3.1.3. Data Preprocessing

In the preprocessing stage of the COVID-19 images, CNN models use annotating lesions for each CT volume in which lung masks are implemented in the training phase to form a mask volume. This mask volume is concatenated with the CT volume to obtain the final CT volume. The final CT volume is then set to a specific resolution (e.g., 200 ∗ 400) to prepare it for DL execution. The number of slices of the image sample is fixed and does not change during the image preprocessing phase (they have a range of 73 to 250 in the testing dataset). In this research, the images of the COVID-19 are collected from different sources, including imaging clinics and existing datasets. The images are captured by different types of equipment and contain different acquisition parameters. As a result, there exist considerable variations in the intensity of the images [18]. However, the proposed CNN models implement two standard preprocessing procedures of resizing and normalization to ensure that the CNN models' generalization is not negatively affected.

(i) Resizing: we need first to acquire a constant dimension because all images in this dataset vary in dimension and resolution (365 ∗ 465 to 1125 ∗ 859 pixels). Subsequently, all the images are scaled to specific pixels based on the corresponding CNN models (e.g., NASNet-Large 331 ∗ 331 pixels and NASNetMobile 224 ∗ 224 pixels).
(ii) Normalization: In the normalization part, to set the scaling limit, we use a precalculated mean subtraction of the ImageNet database to normalize the intensity values [56]. Then we scale the intensity values from [0, 255] to the intensity range of [0, 1] using the min-max normalization formula.
  (1) $$\begin{array}{c} x_{\text{norm}}=\frac{x-x_{\min}}{x_{\max}-x_{\min}}. \end{array}$$

#### 3.1.4. Deep Learning for Feature Extraction

The quality and quantity of the extracted features from images play an important role in producing robust and accurate diagnosis results. The DL CNN requires a much larger number of features and data size to minimize the error of the classification. A small-scale data might cause problems such as imbalanced training and overfitting [57]. The feature extraction of this work is first implicitly performed according to the CNN models' standard architecture, as each model has its own existing feature extraction algorithms. However, to obtain more significant classification results, we need to increase the dimensionality of the features as the COVID-19 dataset considerably has a small number of images. Hence, we implement selected feature extraction algorithms that are suitable for deep convolutional feature representation to produce an additional computed encoded feature vector [58]. The initially computed feature vector of the CNN and the computed encoded feature vector are combined in one final feature vector. The corresponding classifiers use the final feature vector to produce the diagnosis results.

#### 3.1.5. Evaluation Measurements

In this study, we used the most common evaluation metrics, including the area under the curve (AUC), classification accuracy rate (CAR), *F*1-score, receiver operating characteristics (ROC) curve, precision, recall, and mean squared error (MSE). They are calculated based on the classification results of true positive rate (TPR), false positive rate (FPR), predictive positive value (PPV), and negative predictive value (NPV). Accordingly, equations (2) to (6) represent the mathematical description of the evaluation metrics:

(i) Classification Accuracy Rate: It is known as classification accuracy rate (CAR), and the CAR shows how the output results near for the actual outcomes, which is calculated using the following equation:
  (2) $$\begin{array}{c} CAR=\frac{\left(TP+TN\right)}{\left(TP+TN+FP+FN\right)}\times 100. \end{array}$$
(ii) Precision: It is utilized to measure the ability of a classifier to identify the importance of classified subjects and reject insignificant subjects, which is calculated using the following equation:
  (3) $$\begin{array}{c} \text{Precision}=\frac{TP}{TP+FP}. \end{array}$$
(iii) Recall: It is utilized to measure and evaluate the importance level of the classified subjects, which is calculated using the following equation:
  (4) $$\begin{array}{c} \text{Recall}=\frac{TP}{TP+FN}. \end{array}$$
(iv) ROC: The ROC curve is utilized to graphically plot the classifier's overall performance in terms of providing the correct results by plotting the TPR against the FPR.
(v) Mean Absolute Error: The mean absolute error (MAE) is a linear score that is widely used for calculating classification error, which is calculated using the following equation:
  (5) $$\begin{array}{c} \text{MAE}=\frac{1}{N}\sum_{i=1}^{N}\left|y_{i}-{\hat{y}}_{i}\right|. \end{array}$$
(vi) *F*1-score: The *F*1-score is extracted from measuring the precision and recall in which the best *F*1-score has the value of 1 or near to the value of 1 and the worst *F*1-score has the value of 0 or near to the value of 0, which is calculated using the following equation:
  (6) $$\begin{array}{c} F1-\text{score}=\frac{\text{Precision}*\text{Recall}}{\text{Precision}+\text{Recall}}. \end{array}$$

### 3.2. Weighting Stage

The crow swarm optimization (CSO) is used to find the best set of coefficients that can be applied through a designed fitness function to evaluate the performance of the used deep learning algorithms. CSO is designed in a way that will ensure a good distribution for all the selected coefficients, this was done by taking the best available average fitness (not just the best one). In this section, the inspiration of the proposed method and the mathematical model are discussed.

#### 3.2.1. Inspiration

The American crow (*Corvus brachyrhynchos*) is an example of a species that has evolved complicated social behaviors. They are kind of crows, conjointly called the common crow. They are living in North-western yank. The crows are divided into teams, in which the typical cluster size of American crows outbound, their last hunt site of the day was 237 ± 43. They are ready to reach speeds of 35–43 mph. Daytime hunt aggregations of crows throughout the nonbreeding season area unit sometimes composed of various family teams [59]. Yank Crow's kind communal roosts will vary from 100 to 2 million crows [59]. However, these hunt sites' area unit are usually not among the visibility of their roosting sites. American crows' area unit make a superb model species to conduct analysis on social behavior because they prominently forage in teams before sunset and form massive communal roosts in the dark throughout the nonbreeding season [60].

Communal roosts perform as info-sharing centers. At these communal roosts, crows share info like wherever to forage throughout the day. Crows that have not found sensible an honest forage site can follow crows that have found good forage sites the following day [59]. Communal roosts conjointly aid in thermoregulation and predator turning away [42]. The dimensions of the communal roost tend to extend because the weather gets colder. In distinction to their evening communal roosts, American crows are divided into smaller teams to forage throughout the day. Each morning, crows disperse from their communal roosting site and travel up to 40 miles away to forage.

There three predictions that will facilitate support this hypothesis:

- American crows can leave their communal search sites in giant teams, as critical singly.
- American crows can depart their communal forage websites when the sunset and fly along towards their communal roosting site to own the longest forage opportunities day by day.
- American crows can fly within the direction of their communal roosting site once outward their last communal search site.

#### 3.2.2. Mathematical Model and Algorithm

The algorithm of CSO together with its mathematical model is presented in these subsections.

*(1) Group Division*. The CSO algorithmic program mimics the behavior of *Corvus brachyrhynchos*. To model such interactions, every cluster of crows' area unit needed to maneuver over the search area. As mentioned earlier, the crows being divided into teams who begin to look for places of food at long distances area and not among the scope of traditional vision. Assume the crow's algorithmic program determines the simplest cluster you get when choosing the food space and additionally deciding the totals that did not get sensible food on this trip. Within the next journey of food search, teams with dangerous food can eat sensible food. Reckoning on the characteristics of the animal, like speed, angle for departure, and placement. This behavior is delineating by the following equation:

(7) $$\begin{array}{c} S_{i+1}=\left(R*S_{i}\right)+\left(P_{\text{best}}-P_{i}\right)*\mathrm{R,} \end{array}$$

where *i* indicates the current iteration, *R* is a random number between (0,1), **P**best is the position vector of the best solution obtained so far, *P*_*i*_ is the position vector, *S*_*i*_ is the velocity value, the velocity is between (−6, 6).

*(2) Update Position*. The update position for each crow in the group depends on the best crow's position in that group, and this can be done using the following equation:

(8) $$\begin{array}{c} P_{i+1}=P_{i}+S_{i+1}*cos\left(\theta \right), \end{array}$$

where *P*_*i*+1_ is a new position and Ɵ is an angle for departure between (45, 135). The position should be updated in each iteration.

*(3) Update the Angle*. When the best crow follows the behavior, the worst crow angle will be updated according to the following equation:

(9) $$\begin{array}{c} \frac{\theta i+1=\left(\theta i+\theta \mathrm{best}\right)}{2}, \end{array}$$

where Ɵ_*i*+1_ is the new angle for crow, *R* is a random number between (0, 1), Ɵ_*i*_ is the current angle of crow, and Ɵ_best_ is the angle of best crow.

The important stage in the operations of a solution is the initialization process that provides the algorithm needs and the data of the problem and submits it. The preparedness phase consists of several stages. The first phase is the process of reading the problem database information. Thereafter generate several units for all measures. The sum of units must be 100 that are randomly distributed for the nine measures.

In the second stage, we applied the CSO algorithm to solve this problem. It is started by calculating the value of the initial speed and the angle for all crows. In this step, the speed value is between (−6, 6), and the angle value is between (45, 135). This procedure mimics the situation in a real American crow. This case represents the crow's first movement to search for the source of the feed (food). When selecting any path, crows can receive quantities of food. These routes do not necessarily lead to the feed source. Therefore, the food during this case is a guide that works on the ways that are taken by crows and not necessarily the food path. A solution can be constructed using speed, angle, and best position in-group. After the initialization step, the CSO algorithm starts to work. Crows start to move from the beginning node that had been chosen in the initialization stage. The following fitness function is used to evaluate each solution, the problem is formulated as a 2D matrix (15 ∗ 9), as there are 15 algorithms to be evaluated with nine measures, and the goal of the proposed fitness equation is to find the overall performance for each one of 15 algorithms.

(10) $$\begin{array}{c} \text{Fitnees}\left(i\right)=x1*\text{AUC}\left(i\right)+x2*\text{CAR}\left(i\right)+x3*F\text{Score}\left(i\right)+x4*\text{Precision}\left(i\right)+x5*\text{Recall}\left(i\right)\\ +-x6*\text{FPR}\left(i\right)+x7*\text{PPV}\left(i\right)+x8*\text{NPV}\left(i\right)-x9*\text{MSE}\left(i\right). \end{array}$$

We update position (number of units) depending on the previous position, speed, and crow angle. Before updating the position, the speed must be updated depending on the previous speed, which is different between the positions of the best crow and the current crow. The third stage is the updated angle for every crow. Lastly, after several iterations, we returned the best average for all students and distributed the units for the classifier. Pseudocode of CSO is presented in Algorithm 2.

where *i* indicates the current iteration, *R* is a random number between (0, 1), *P*_best_ is the position vector of the best solution obtained so far, *P*_*i*_ is the position vector, *S*_*i*_ is the velocity value, the velocity is between (−6, 6). *P*_*i*+1_ is a new position, and Ɵ is an angle for departure between (45,135). Ɵ_*i*+1_ is the new angle for crow, *R* is a random number between (0, 1), Ɵ_*i*_ is the current angle of crow, and Ɵ_best_ is the best crow angle. The position should be updated in each iteration.

#### 3.2.3. CSO Benchmarking with Other Swarm Optimization Algorithms

CSO algorithm is evaluated by using 30 benchmark functions. Some of those functions are standard functions that are used in researches. These functions are chosen to be able to show the performance of CSO and to compare it with some known algorithms. The selected 30 test functions are shown in Tables 3 and 4, where *D* means the function's dimension, range means the function's search space limits, and Opt is the optimal value. The selected functions are unimodal or multimodal benchmark minimization functions. Unimodal test functions have a single optimum value; thus, they can benchmark an algorithm's convergence and exploitation. Multimodal test functions have more than one optimum value, making them more challenging than unimodal. An algorithm should avoid all the local optima to approach and approximate the global optimum. So, exploration and local optima avoidance of algorithms can be benchmarked by multimodal test functions.

For each benchmark function, the CSO algorithm and the compared algorithms are performed in the experiments under the condition of the same number of iterations (1000), independent runs for 30 times, and the population size is set to 50. The statistical results (average and standard deviation) are shown in Tables 5 and 6. For verifying the results, the CSO algorithm is compared with GWO [61], HHO [62], SSA [63], and WOA [64].

The results in Table 5 demonstrated that CSO is better than the selected algorithms in most unimodal (nine out of 15) test functions. Unimodal functions test the exploitation of an algorithm. The obtained results showed CSO superiority in exploiting the optimal value, so CSO provides excellent exploitation ability.

For testing the exploration strength of an algorithm, the multimodal functions are used as the number growing exponentially with dimension such types of functions. The results in Table 6 demonstrated that CSO is better than the selected algorithms on most (13 out of 15) multimodal functions. The obtained results show the superiority of the CSO algorithm in terms of exploration. Algorithms' average fitness on the test functions is presented in Figure 3, and the standard deviations of the algorithms on the test functions are shown in Figure 4.

### 3.3. Selection Stage

In this stage, among 15 deep learning models, the final diagnostic model will be selected based on evaluation experiment with CSO benchmarked algorithm. Furthermore, the winner model is the one that achieved best results in all evaluation measurements without presenting any overfitting or underfitting classification performance in all classes.

## 4. Results and Discussion

### 4.1. Results of Evaluation Stage

To the best of the authors' knowledge, this was the first study to carry out supervised COVID-19 identification with large numbers of CT cases within the cutting-edge healing center during the current COVID-19 pandemic through developing and training a successful deep learning model on collected Lung CT samples. The study's motivation is to utilize AI to lighten the issue of proficient interpretation deficiencies for CT lung scan when the virus is still spreading rapidly. Although there were numerous viable AI uses in past works [7], improving AI for automated COVID-19 identification is still challenging. First, the number of patients registered is moderately littler within the current crisis circumstance than in past works [2, 27]. The patients selected in our research are clinically analyzed with COVID-19 as most of the patients did not experience PCR testing due to an unexpected outbreak and limited therapeutic resources in a limited time. Second, radiologists did not label COVID-19 samples in CT lung scan regions and labeled COVID-19 samples for the patients can be classified (COVID-19 or healthy) to train the deep learning models in this research. Third, the proficient radiologist may miss a few tiny infected regions of COVID-19, and it remains unclear whether deep learning-based models can be detected. We hypothesized solving these problems by offering delicate deep learning models, that is, ResNet50, GoogleNet, and MobileNetV2. The first problem is solved using broad CT lung training samples to get perfect training accuracy. Considering the COVID-19 pandemic, the supervised learning issue is used for the second problem [29, 43], such as COVID-19 detection without explaining COVID-19 lesion areas. In this study, the temporally global pooling layer and spatially global pooling layer are utilized in the ResNet50 model to technically handle the COVID-19 identification issue. Finally, to address the third problem by taking advantage of deep learning models and using pretrained CNN models to provide lung masks to guide ResNet50, GoogleNet, and MobileNetV2 learning.

Diagnostic imaging techniques, such as chest radiography and CT, play a significant role in verifying the primary diagnosis of the polymerase chain reaction (PCR) test for COVID-19. Clinical imaging frequently plays a vital role in tracking disease development and patient treatment. Extracting features from radiology modes is an important step in developing profound education models as model success depends directly on the features. This research aims to present an exhaustive study on the classification of COVID-19 in CT imaging using state-of-the-art deep CNN architectures extracted from features and trained in machine learning algorithms based on deep learning models' successful computer vision. The 3-fold cross-validation technology was developed to evaluate each experiment's average classifier generalization performance. For all CNNs, network weights from the weights trained in ImageNet have been initialized. The computer system used in this project, based on Windows, included an Intel(R) Core (TM) i7-8700K 3.7 GHz processor with 32 GB RAM. Python has introduced the training and testing phase of the proposed architecture using a Tens row backend kit as a deep learning application backend, using an 11 GB RAM, NVidia GeForce GTX 1080 Ti GPU.

Popular pretrained and typical models such as ResNet50, DarkNet, GoogleNet, MobileNetV2, Xception, VGG19, VGG16, InceptionV3, ResNet34, CNNs, DNN, SAE, InceptionResNetV2, LSTM, and NASNet-Large models have been trained and tested on CT lung images. The training accuracy and loss values for fold-3 of the pretrained models are shown in Figures 5 and 6, respectively.

The training stage was carried out until the 30th epoch to prevent overfitting for all pretrained models. The diagnostic model's performance outcomes from various pretrained CNN and deep models are in Table 7.

The COVID-19 diagnostic-based deep learning models used in our research are successful compared to recent deep learning computer-aided diagnostic approaches. The deep learning models for 746 CT cases were trained to predict the COVID-19 risks and its influence for early prediction [13]. The deep learning model of 746 lung CT scans was trained for essential lung CT findings [23], and the ROC AUC metric was obtained of 0.92. In our analysis, the 522 scans only are utilized for training tasks; on the other hand, the ROC AUC metric is obtained of 0.90. Based on the variation in the dataset and compared with deep learning models, it was conceivable to identify that classifying COVID-19 can be more straightforward, and the proposed deep learning models are exceptionally effective. As for the incorrect 12 false negative predicted cases, after rechecking the original CT lung cases, the reasons are as follows: there is a slight increase in CT lung regions, and the CT cases of this ground-glass ambiguity are fragile without integration process.

Our research aims to provide a good and promising solution for improving medical diagnostic approaches based on AI for urgent diseases like the COVID-19 pandemic. In addition, to improve the identification, the approach is utilized as a helpful instrument to assist the specialists within the health and medical centers to choose which ideal deep learning model could be used for COVID-19 identification by assessing distinctive deep learning models. The COVID-19 diagnostic deep learning-based models entail the CT lung scan within the current austere battle against this pandemic. However, doctors in hospitals and medical centers are busy treating many COVID-19 patients, and it may be hard for them to do the CT scan for all patients. In this study, the supervised deep learning method provides the location of pulmonary in CT lung lesions.

The annotation attempts of radiologists can be reduced, such as just the provision of COVID-19 classification as a healthy or COVID-19 case. As a result, developing a useful AI instrument has quickly become potential and accessible in clinical applications. In the future, automatic deep learning could significantly reduce the burden on AI experts. The training accuracy and loss values for fold-3 of the pretrained models are shown in Figures 7 and 8, respectively.

The training stage was carried out until the 30th epoch to prevent overfitting for all pretrained models. The diagnostic model's performance outcomes from various pretrained CNN and deep models are presented in Table 8.

### 4.2. Results of Weighting Stage

The COVID-19 optimization method has two significant benefits over other related approaches. Firstly, the input parameters were known defined by disease statistics, stopping scientists from initializing them with random values. Second, the approach can end after several iterations without setting this value. Infected populations initially increase exponentially, but the number of infected people declines after some iterations. The algorithm is executed ten times, and the average results are taken to avoid any randomness in taking the best result only. The ten runs and their average results are shown in Table 9 for the first and second datasets. Each value in the last row of each dataset represents the average of the ten results of each measure. The fitness function uses these averages to get the final performance for each algorithm.

Subsequently, the final result column in the first dataset of Table 10 is obtained by applying equation (10) (fitness function). The values of *x*1 to *x*9 are the average values taken from the last row in Table 9. The average values for the 15 algorithms are shown in Table 10 for the first and second datasets, respectively. The final result represents each deep learning algorithm's overall strength (assessment). The results of the first dataset in Table 10 showed that the ResNet50 algorithm is the best-selected algorithm, and it is of close performance to GoogleNet and LSTM algorithms. InceptionV3 came last as it got the worst overall performance, while the results of the second dataset in Table 10 showed that the VGG16 algorithm is the best-selected algorithm, and it is of close performance to the ResNet50 algorithm. InceptionV3 came last as it got the worst overall performance.

In the first dataset, the ResNet50 algorithm has the highest score of AUC 1317.770678, CAR 1404.603748, *F1*-score 1017.648389, precision 936.6420965, recall 824.2043559, FPR 711.7677382, PPV 537.504169, NPV 390.2033404, and final result 5715.987691. The final results represent the summation of all criteria results and subtracting the MSE. The second-best score is achieved by the GoogleNet algorithm and the InceptionV3 algorithm has the lowest scores among the 15 algorithms. In the second dataset, the VGG16 algorithm has the highest score of AUC 1299.884286, CAR 1302.852674, *F1*-score 1143.826591, precision 1036.285298, recall 735.858182, FPR 664.348122, PPV 465.3038828, NPV 439.9139883, MSE 0.785912024 (lowest), and final result 5758.790868. The second-best score is achieved by the ResNet50 algorithm and the InceptionV3 algorithm also has the lowest scores among the 15 algorithms. Our analysis is an optimized combination of 10 tests and 15 deep learning methods for COVID-19 identification. The crow swarm optimization (CSO) is used to find the best set of coefficients that can be applied through a designed fitness function to evaluate the performance of the used deep learning algorithms. CSO is designed to ensure a good distribution for all the selected coefficients. This operation took the best available average fitness (not just the best one). The CSO algorithm is utilized to assess the diverse deep learning approaches for COVID-19 regarding the assessment measures. The research outcomes revealed that the selection problem related to COVID-19 identification methods could be viably solved utilizing the CSO approach.

This work concerns with early classification of COVID-19 as it is important for the treatment and control of diseases. Compared to reverse transcription-polymerase chain reaction (RT-PCR), chest computed tomography (CT) imaging can be a much more accurate, effective, and rapid technique for classifying and assessing COVID-19, especially in the pandemic area. Almost all hospitals have CT imaging machines; thus, CT images in the chest can be used for the early diagnosis of COVID-19 patients. The CT-based chest diagnosis of COVID-19 requires a specialist in radiology and a substantial amount of time, which is useful when the outbreak of COVID-19 is through at a rapid rate. Automated analysis of chest CT images is therefore desirable to save the precious time of medical professionals. In the meantime, for predicting cases of COVID-19, several deep learning models have been suggested. There is a need for a choice solution for the optimized COVID-19 deep learning models, which was considered the key issue. In addition, there is no single study to address the issue of optimizing the COVID-19 diagnostic model based on pretrained and trained CNN and in-depth learning. Nevertheless, our research proposed an intellectual framework to assist medical centers and hospitals in selecting the COVID-19 diagnostic model. The assessment of identification approaches for COVID-19 is not a trivial task. Multiple measurements must be evaluated, and some of the measures conflicted with each other.

Our study is mainly constrained by the limitations of the available COVID-19 datasets. As explored in the related studies, the deep learning models need a high and large number of CT lung samples. The selection approach for optimal deep learning COVID-19 diagnostic model based on a novel CSO algorithm can be used for solving complex cases of different related studies to find optimal models. In future directions, the following aspects must be considered to enhance the outcomes of COVID-19 diagnostics: first, suggest to use more trained deep learning models that help evaluate and select the proposed approach for optimal deep learning COVID-19 diagnostic model based on a novel CSO algorithm. Second, using more measurements to support and evaluate the selection approach for optimal deep learning COVID-19 diagnostic model based on a novel CSO algorithm. In addition, the main limitation of the CSO algorithm, like all swarm algorithms, is no guarantee to find the optimal solution. This is due to the nature of the problem search space.

## 5. Conclusion

Because of the COVID-19 pandemic, the number of computerized COVID-19 diagnosis studies is growing rapidly. This raises the question of which decision-makers should select the optimal COVID-19 diagnostic system in healthcare organizations and which performance criteria should be considered. Because of this, a selection scheme is necessary to address all the above issues. This study aims to bridge the gap between COVID-19 diagnostic model and deep learning models. To the best of the authors' knowledge, there is no work addressed and investigated the selection of the optimal COVID-19 diagnosis models. Only a review of main evaluation measurements for diagnostic COVID-19 deep learning-based models is presented in the scientific literature without addressing bridging the gap between the deep learning models and selection strategy for the optimal model. The crow swarm optimization (CSO) is employed to find an optimal set of coefficients using a designed fitness function for evaluating the performance of the deep learning model. The CSO is modified to obtain a well-selected coefficient distribution by considering the best average fitness. In this study, we present a description of the mechanism of the proposed methodology development. The outcomes that integrated a mix of 15 deep learning-based methods for COVID-19 diagnosis and nine evaluation metrics are presented in this article. Despite some challenges, including that no similar mechanism has been used to identify the significance of evaluation metrics ranking the deep learning-based models concerning different evaluation metrics is not an easy task, especially considering that some metrics conflict with each other. Our work will address all the challenges when developing the integrated framework. With a massive number of COVID-19 diagnostic deep learning-based models, it is not a trivial task for healthcare managers to decide which model meets their requirements with respect to reliability, cost, and speed. This is the main challenge of our study. The CSO algorithm is utilized to assess the diverse deep learning approaches for COVID-19 regarding the assessment measures. The research outcomes revealed that the selection problem related to COVID-19 identification methods could be viably solved utilizing the CSO optimization approach. For the first dataset, the ResNet50 algorithm is the optimal deep learning model is selected as the ideal identification approach for COVID-19 with the closeness overall fitness value of 5715.988 for COVID-19 CT lung images case considered differential advancement. In contrast, the VGG16 algorithm is the optimal deep learning model. It is selected as the ideal identification approach for COVID-19 with the closeness overall fitness value of 5758.791 for the second dataset. Furthermore, selecting an inappropriate COVID-19 diagnostic model might be non-cost effective for medical and health institutions with a strong need for a rapid and accurate diagnostic model. Our proposed methodology will help healthcare managers assess and evaluate the COVID-19 diagnostic model and select the optimal model that fits their requirements by saving time, cost, and effort and obtain accurate and reliable results. Our proposed methodology can be used to evaluate a diagnostic model that uses the chest X-ray image to assist healthcare administrators in deciding which is the best COVID-19 diagnostic model.

## Figures and Tables

**Figure 1:** The selection approach for optimal deep learning COVID-19 diagnostic model based on novel CSO algorithm.

**Figure 2:** COVID-19 CT lung scan cases.

**Figure 3:** The average fitness of the algorithms on the test functions.

**Figure 4:** The standard deviations of the algorithms on the test functions.

**Figure 5:** First dataset training accuracy for ResNet50 model.

**Figure 6:** First dataset loss values for ResNet50 model.

**Figure 7:** Second dataset training accuracy for ResNet50 model.

**Figure 8:** Second dataset loss values for ResNet50 model.

**Algorithm 1:** Pseudocode for the selection approach for optimal deep learning COVID-19 diagnostic model based on novel CSO algorithm.

**Algorithm 2:** Pseudocode of CSO.

**Table 1:** Deep learning models.

No.	DL model	Description	Remark
1.	CNN	It consists of a set of fully connected layers and convolution layers	Require a few input parameters
2.	DarkNet	Classification model for object detection	Used for real-time object detection
3.	DNN	It has many hidden nodes compared with the conventional neural network	Performs deep nonlinear analysis
4.	GoogleNet	It is an improved DL model for image analysis	Used for object detection with a few input parameters
5.	InceptionResNetV2	It has a fixable architecture of a CNN	Used for different types of applications
6.	Inceptionv3	Third generation of Google's Inception CNN	Used for classifying visual objects for computer vision applications
7.	LSTM	A type of recurrent neural network (RNN)	Used for dealing with sequences of data
8.	MobileNetV2	A lower complexity and model size DL neural network proposed by Google for mobile phone image processing applications	Used for object detection, classification, and semantic segmentation
9.	NASNet-Large	A CNN modeled to deal with a large scale of image datasets.	Used to classify objects
10.	ResNet34	A CNN architecture but with shortcuts and bottleneck block mechanisms between layers to speed up solving problems.	Used for deep real-time analysis
11.	ResNet50	A type of CNN that performs deeper analysis to solve complex problems	The deeper analysis might degrade the accuracy of the network
12.	SAE	A multilayer neural network with a stacked autoencoder	Used for datasets with a small dimension of features.
13.	VGG16	A CNN with multiple 3 × 3 kernel-sized filters in the convolutional layers	Used for recognition tasks of a large-scale number of images dataset
14.	VGG19	A CNN with multiple 3 × 3 kernel-sized filters in the convolutional layers with additional layers than the VGG16	Used for recognition tasks of a large-scale number of images dataset
15.	Xception	An improved version of the Inception family of CNN	Used for classifying visual objects for computer vision applications with a slightly higher accuracy

**Table 2:** Parameters of the COVID-19 deep learning models.

Model no.	Deep learning model	Tuning parameters
1	CNN	Momentum = 0.5 to 0.9; number of epochs = 0.9; batch size = 32.
2	DarkNet	batch = 64; momentum = 0.9; learning_rate = 0.000008.
3	DNN	batch_size = *c* (32, 64), dropout_rate = *c* (0.1, 0.2, 0.3), units = *c* (10, 20).
4	GoogleNet	Each one must be resized from 647 × 511 × 3 to 227 × 227 × 3 pixels, the dimensions used to train GoogleNet 224 × 224 × 3 pixels.
5	InceptionResNetV2	Outputs = Dense (100, activation = 'softmax') (base_model.output) model = Model (base_model.inputs, outputs).
6	Inceptionv3	batch_size = *c* 64, dropout_rate = *c*(0.1, 0.2, 0.3), units = *c* (10,20, 30).
7	LSTM	Rule search (evaluation measure) = entropy; minimum rule coverage = 2, maximum rule length = 6.
8	MobileNetV2	learning_rate = 0.0001; no. of epochs = 10.
9	NASNet-large	learning_rate = 0.0002; no. of epochs = 20.
10	ResNet34	Optimization method: Adam; momentum: 0.90; weight-decay: 0.0006; dropout: 0.6; batch size: 100; learning rate: 0.02; total no. of epochs: 20.
11	ResNet50	Optimization method: Adam; momentum: 0.97; weight-decay: 0.0005; dropout: 0.7; batch size: 100; learning rate: 0.03; total no. of epochs: 30.
12	SAE	batch_size = *c* (64), dropout_rate = *c* (0.1, 0.2, 0.4), units = *c* (10, 20, 40).
13	VGG16	Optimization method: SGD; momentum: 0.90; weight-decay: 0.0004; dropout: 0.6; batch size: 164; learning rate: 0.06; total no. of epochs: 60.
14	VGG19	Optimization method: SGD; momentum: 0.97; weight-decay: 0.0005; dropout: 0.3; batch size: 128; learning rate: 0.07; total no. of epochs: 40.
15	Xception	Optimizer method: SGD; momentum: 0.8; learning rate: 0.035; learning rate decay: decay of rate 0.92 every 4 epochs.

**Table 3:** Unimodal benchmark functions.

Function	Equation	Test name	*D*	Range	Opt
F1	*f*_1_(*x*)=*∑*_*i*=1_^*n*^*x*_*i*_^2^	Sphere	30	−100, 100	0
F2	*f*_2_(*x*)=*∑*_*i*=1_^*n*^|*x*_*i*_|+*∏*_*i*=1_^*n*^|*x*_*i*_|	Schwefel 2.22	2	−100, 100	0
F3	*f*_3_(*x*)=max_*i*_{|*x*_*i*_|, 1 ≤ *i* ≤ *n*}	Schwefel 2.21	2	−100, 100	0
F4	*f*_31_(*x*)=2*x*_1_^2^ − 1.05*x*_1_^4^+*x*_1_^6^/6+*x*_1_*x*_2_+*x*_2_^2^	Three-Hump Camel	2	−5, 5	0
F5	$f_{6}\left(x,y\right)=-200e\sqrt[{-0.2}]{x^{2}+y^{2}}$	Ackley 2	2	−32, 32	−200
F6	*f*_7_(*x*)=*x*_1_^2^+*x*_2_^2^ − 0.3 cos(3*πx*_1_) − 0.4 cos(4*πx*_2_)+0.7	Bohachevskyn N.1	2	−100, 100	0
F7	*f*_8_(*x*) =(*x*_1_ + 2*x*_2_ − 7)^2^+(2 *x*_1_ +*x*^2^ −5)^2^	Booth	2	−10, 10	0
F8	*f*_38_(*x*)=−*∑*_*i*=1_^*d*^(*x*_*i*_ − 1)^2^ − *∑*_*i*=2_^*d*^*x*_*i*_*x*_*i*−1_	Trid	6	−36, 36	−50
F9	*f*_9_(*x*)=*∑*_*i*=1_^*n*^*x*_*i*_^2^+(*∑*_*i*=1_^*n*^0.5*ix*_*i*_)^2^+(*∑*_*i*=1_^*n*^0.5*ix*_*i*_)^4^	Zakharov	2	−5.12, 5.12	0
F10	$f\left(x\right)-1+\cos\left(\sqrt[{12}]{x_{1}^{2}+x_{2}^{2}}\right)/0.5\left(x_{1}^{2}+x_{2}^{2}\right)+2$	Drop Wave	2	−4.5, 4.5	−1
F11	*f*_13_(*x*) = *∑*_*i*=1_^*n*^*x*_*i*_^10^	Schwefel 2.23	2	−100, 100	0
F12	*f*_14_(*x*) = *∑*_*i*=1_^*n*^*|x*_*i*_	Schwefel 2.20	2	−100, 100	0
F13	*f*_18_(*x*)=*∑*_*i*=1_^*d*/4^[(*x*_4*i*−3_+10*x*_4*i*−2_)^2^+5(*x*_4*i*−1_+*x*_4*i*_)^2^+(*x*_4*i*−2_+*x*_4*i*−1_)^4^+10(*x*_4*i*−3_+*x*_4*i*_)^4^]	Powell	10	−4, 5	0
F14	*f*_19_(*x*)=*∑*_*i*=1_^*d*^[(*∑*_*j*=1_^*d*^*x*_*j*_^*i*^)*b*_*i*_]^2^	PowerSum	4	0, 4	0
F15	*f*_4_(*x*) = *∑*_*i*=1_^*n*^[*b*(*x*_*i*+1_ − *x*_*i*_^2^)^2^+(*a* − *x*_*i*_)^2^]	Rosenbrock	30	−2.048, 2.048	0

**Table 4:** Multimodal benchmark functions.

Function	Equation	Type	Test name	D	Range	Opt
F16	$f_{20}\left(x\right)=-20\;\exp\left(\sqrt[{-0.2}]{\sum_{i=1}^{n}x_{i}^{2}}\right)-\exp\left(1/n\sum_{i=1}^{n}\cos\left(2\pi x_{i}\right)\right)+20+e$	N	Ackley	2	−10, 10	0
F17	*f*_22_(*x*)=*∑*_*i*=1_^*n*^*ix*_*i*_^4^+random[]0,1)	N	Quartic	10	−1.28, 1.28	0+rand
F18	*f*_23_(*x*) = (4–2.1 *x*_1_^2^ + *x*_1_^4^/3) *x*_1_^2^ + *x*_1_*x*_2_ +(−4+4 *x*_2_^2^) *x*_2_^2^	N	Six-Hump Camel	2	−5, 5	−1.0316
F19	*f*_24_(*x*) = *a* (*x*_2_ - *bx*_1_^2^ + *cx*_1_ – *r*)^2^ + *s*(1- *t*) cos(*x*_1_) + *s*		Branin	2	−5, 15	0.3979
F20	*f*_25_(*x*) = [1 + (*x*_1_ + *x*_2_ + 1)^2^ (19 – 14 *x*_1_ + 3*x*_1_^2^ − 14 *x*_2_ + 6 *x*_1_*x*_2_ + 3*x*_2_^2^)] ∗ [30 + (2*x*_1_ + 3 *x*_2_)^2^ (18 – 32 *x*_1_ + 12*x*_1_^2^ − 48 *x*_2_ + 36 *x*_1_*x*_2_ + 27*x*_2_^2^)]	N	Goldstein Price	2	−2, 2	3
F21	*f*_26_(*x*)=−*∑*_*i*=1_^4^*c*_*i*_exp(−*∑*_*j*=1_^3^*a*_*ij*_(*x*_*j*_ − *p*_*ij*_)^2^)	F	Hartmann 3-D	3	1, 0	−3.8628
F22	*f*_27_(*x*)=−*∑*_*i*=1_^4^*c*_*i*_exp(−*∑*_*j*=1_^6^*a*_*ij*_(*x*_*j*_ − *p*_*ij*_)^2^)	F	Hartmann 6-D	6	1, 0	−3.3224
F23	$f_{32}\left(x\right)=\;-200\;e^{-0.2\sqrt{x^{2}+y^{2}}}$ + 5 *e*^cos(3*x*)+sin(3*y*)^		Ackley 3	2	−32, 32	−195.629
F24	*f*_33_(*x*)=*x*_1_^2^+2*x*_2_^2^ − 0.3 cos(3*πx*_1_)cos(4*πx*_2_)+0.3	N	Bohachevskyn N.2	2	−10, 10	0
F25	*f*_34_(*x*)=sin(*x*)*e*^(1 − cos(*y*))^2^^ + cos(*x*)*e*^(1 − sin(*x*))^2^^ + (*x* − *y*)^2^	N	Brid	2	−2pi, 2pi	−106.7645
F26	$f_{35}\left(x\right)={\left(\left|\sin\left(x_{1}\right)\sin\left(x_{2}\right)\exp\left(\left|100-\sqrt{x_{1}^{2}+x_{2}^{2}}/\pi \right|\right)\right|+1\right)}^{0.1}$	N	Cross in Tiny	2	−10, 10	−2.06261
F27	*f*_36_(*x*)=−cos(*x*_1_)cos(*x*_2_)exp(−(*x*_1_ − *π*)^2^ − (*x*_2_ − *π*)^2^)	F	Easom	2	−100, 100	−1
F28	$f_{37}\left(x\right)=-\sin^{2}\;\left(x-y\right)\;\;\sin^{2}\;\left(x+y\right)/\sqrt{\left(x^{2}+\;y^{2}\right)}$	N	Keane	2	0, 10	−0.6737
F29	$f_{41}\left(x\right)=-\left|\sin\left(x_{1}\right)\exp\left(\left|1-\sqrt{x_{1}^{2}+\;x_{2}^{2}}/\pi \right|\right)\right|$	N	Holder	2	−10, 10	−19.2085
F30	*f*_43_(*x*)=−*∑*_*i*=1_^*d*^sin(*x*_*i*_) sin^2m^(*ix*_*i*_^2^/*π*)	N	Michalewics	2	1.57, 2.21	−1.8013

**Table 5:** Unimodal benchmark functions.

Name	CSO		GWO		HHO	
	AV	STD	AV	STD	AV	STD
Sphere	1.10132*E* − 12	2.17067*E* − 12	8.32056*E* − 62	2.01043*E* − 61	5.75505*E* − 96	1.21415*E* − 95
Schwefel 2.22	5.5237*E* − 112	1.5496*E* − 111	8.74*E* − 99	0	1.11321*E* − 48	1.51435*E* − 48
Schwefel 2.21	1.4406*E* − 111	6.7475*E* − 111	1.26*E* − 105	0	2.95204*E* − 51	6.83343*E* − 51
Camel3	0	0	0	0	1.1048*E* − 107	2.3653*E* − 107
Ackley2	−200	0	−200	0	−200	0
Bohachevskyn N. 1	0	0	0	0	0	0
Booth	0	0	1.54098*E* − 07	1.11392*E* − 07	2.36488*E* − 05	2.5515*E* − 05
Trid	−50	0	−49.99989	8.03012*E* − 05	−1367.28225	4.374233259
Zakharov	7.9142*E* − 221	0	0	0	9.5294*E* − 47	2.13084*E* − 46
Drop Wave	−0.98496333	0.027373716	−0.99574666	0.016186579	−1	0
Schwefel 2.23	0	0	0	0	0	0
Schwefel 2.20	1.0876*E* − 111	5.4846*E* − 111	3.21*E* − 88	0	3.48466*E* − 47	4.72514*E* − 47
Powell	0.001705466	0.001128045	4.94865*E* − 07	6.09827*E* − 07	4.9489*E* − 104	7.662*E* − 104
PowerSum	0.051633374	0.070129514	0.106802381	0.261322987	1.4218*E* − 131	2.4194*E* − 131
Rosenbrock	7.610173333	21.01106746	26.74104667	0.704408086	0.008242153	0.010289518

**Table 6:** Multimodal benchmark functions.

Name	CSO		GWO		HHO	
	AV	STD	AV	STD	AV	STD
Ackley	8.8818*E* − 16	4.01173*E* − 31	8.8818*E* − 16	4.01173*E* − 31	−8.8818*E* − 16	0
Quartic	0.031253333	0.018374115	0.000971688	0.000902519	0.000445553	0.000297211
6-Hump Camel	−1.0316	6.77522*E* − 16	−1.031628448	4.31084*E* − 09	−1.0316	0
Branin	0.3979	0	0.397887852	5.97628*E* − 07	0.397946667	9.81495*E* − 05
Goldstein	3	0	3.000007881	9.28286*E* − 06	3	0
Hart3	−3.8628	3.16177*E* − 15	−3.8620812	0.001938044	−3.854683333	0.008125864
Hert6	−3.3224	1.35504*E* − 15	−3.264253912	0.099876517	−2.9311	0.07435459
Ackley3	−195.629	5.78152*E* − 14	−195.6290282	2.8506*E* − 08	−186.4112	0
Bohachevskyn N. 2	0	0	0	0	0	0
Bird	−106.7645	7.2269*E* − 14	−106.1160683	3.551734418	−106.7645	−106.7645
Cross_in_Tiny	−2.06261	0	−2.062611869	3.30268*E* − 09	−2.0626	0
Easom	−1	0	−1	0	−0.99998	8.16497*E* − 06
Keane	−0.6737	1.1292*E* − 16	−0.6737	1.1292*E* − 16	−0.67367	0
Holder	−19.2085	3.61345*E* − 15	−19.20849251	8.17787*E* − 06	−19.2085	0
Michalewics	−1.8013	6.77522*E* − 16	−1.8013	6.77522*E* − 16	−1.8013	0

**Table 7:** The first dataset diagnostic performance outcomes of various pretrained models.

No	Classifier	AUC	CAR	*F1*-score	Precision	Recall	FPR	PPV	NPV	MSE
1	ResNet50	90.78	91.46	90.49	89.73	88.94	90.92	90.22	90.17	0.039
2	DarkNet	80.92	85.13	85.11	83.29	80.14	82.19	83.71	81.95	0.069
3	GoogleNet	86.99	90.35	89.42	90.21	90.11	88.92	90.47	90.16	0.044
4	MobileNetV2	85.47	88.36	87.69	83.33	86.91	82.14	85.25	86.94	0.038
5	Xception	75.14	77.13	75.02	76.96	74.82	77.37	74.38	72.96	0.094
6	VGG19	80.32	84.38	84.29	77.43	93.56	82.14	83.64	81.79	0.081
7	VGG16	81.36	80.14	80.25	78.97	79.46	78.19	80.03	76.91	0.078
8	InceptionV3	63.40	65.98	64.81	66.47	64.91	62.99	65.11	63.73	0.055
9	ResNet34	90.54	90.71	80.48	79.28	80.10	89.79	90.21	89.94	0.042
10	CNNs	87.47	88.15	83.36	87.55	87.89	86.36	87.99	86.69	0.057
11	DNN	83.39	85.36	81.30	83.57	85.66	83.96	84.14	82.64	0.063
12	SAE	80.39	82.14	79.92	84.87	81.93	80.97	83.94	83.12	0.059
13	InceptionResNetV2	85.67	87.95	86.11	87.64	84.24	86.14	88.19	85.37	0.098
14	LSTM	88.25	90.54	88.36	89.25	88.97	86.91	90.11	87.67	0.096
15	NASNet-Large	79.36	80.11	78.98	77.91	78.16	75.87	79.47	82.96	0.079

**Table 8:** The first dataset diagnostic performance outcomes of various pretrained models.

No	Classifier	AUC	CAR	*F1*-score	Precision	Recall	FPR	PPV	NPV	MSE
1	ResNet50	90.89	89.10	87.23	88.63	87.74	88.93	88.75	90.33	0.054
2	DarkNet	82.22	84.23	83.45	82.27	82.34	84.16	83.21	82.44	0.075
3	GoogleNet	84.76	86.76	84.91	85.20	85.10	85.72	83.33	84.36	0.059
4	MobileNetV2	83.12	85.33	84.19	84.37	83.49	84.87	85.10	83.22	0.047
5	Xception	84.83	81.35	80.12	79.99	80.43	80.84	80.32	80.98	0.061
6	VGG19	84.22	84.97	84.77	82.46	82.86	83.33	83.47	81.23	0.046
7	VGG16	91.34	89.96	88.75	88.15	88.95	88.97	89.14	87.99	0.038
8	InceptionV3	72.21	75.34	73.81	73.47	73.83	74.87	72.34	74.84	0.069
9	ResNet34	90.42	88.21	86.48	82.97	87.22	87.53	87.39	76.27	0.048
10	CNNs	85.29	83.65	83.10	82.55	81.76	82.40	82.77	82.74	0.050
11	DNN	81.96	83.50	82.37	83.12	82.12	83.12	81.94	82.84	0.083
12	SAE	83.10	82.90	81.87	80.43	81.27	81.84	81.36	81.38	0.078
13	InceptionResNetV2	88.38	88.35	87.43	86.76	86.42	87.53	88.05	87.46	0.069
14	LSTM	82.44	83.24	82.33	82.58	83.09	82.77	82.55	79.24	0.099
15	NASNet-Large	81.11	82.35	80.48	80.21	80.68	81.31	81.68	82.16	0.062

**Table 9:** CSO results for 10 runs.

Fitness	AUC	CAR	*F1*-score	Precision	Recall	FPR	PPV	NPV	MSE	Speed	Angle
*The results of the first dataset*											
71.82	14.45	17.46	10.59	8.50	10.16	9.63	5.72	5.19	18.28	0.69	53
81.32	14.76	12.38	17.45	9.11	10.53	6.66	5.77	3.49	19.81	0.77	129
77.12	14.26	18.53	13.51	7.51	9.96	8.46	6.05	3.42	18.27	−3.43	53
70.41	13.72	16.09	9.28	7.80	9.46	9.49	6.76	5.36	22.02	−2.22	45
77.73	14.30	18.10	11.57	12.52	6.01	6.87	4.06	4.13	22.42	−2.08	131
72.54	14.32	18.19	8.71	12.45	11.10	8.41	4.04	4.16	18.58	3.89	59
73.34	13.85	11.17	10.51	10.37	8.70	8.18	6.76	3.92	26.51	−3.31	57
73.57	15.19	11.23	10.65	9.18	9.31	7.60	8.09	6.78	21.94	3.99	67
78.56	14.73	17.97	9.035	13.52	10.27	5.60	6.08	3.17	19.60	2.46	57
76.20	15.55	12.41	11.11	13.38	7.11	7.33	6.25	3.65	23.17	−2.92	48
75.26	14.51	15.35	11.24	10.43	9.26	7.82	5.96	4.33	21.06	−0.21	69.9

*The results of the second dataset*											
74.26	14.18	14.50	12.00	9.93	10.21	8.70	5.11	5.50	19.85	3.71	57
79.03	13.89	12.48	13.01	14.99	9.42	5.79	4.54	6.00	19.86	2.08	46
74.31	14.15	18.68	12.20	11.80	7.76	7.64	5.38	5.44	16.93	−5.67	112
74.45	14.02	18.21	10.04	10.04	6.37	7.35	4.50	4.77	24.68	2.42	110
80.88	14.04	17.33	15.03	12.88	8.79	6.03	3.88	4.60	17.41	−0.02	56
81.85	14.19	11.93	15.54	12.34	7.44	4.91	7.71	5.72	20.20	−0.19	54
81.90	14.26	12.50	15.55	14.38	5.48	5.69	6.01	3.97	22.16	4.91	45
71.74	14.70	11.93	10.40	9.13	10.66	8.85	6.53	6.15	21.62	−2.16	87
73.61	13.37	11.87	13.22	9.56	10.16	10.21	4.09	4.20	23.31	−3.03	58
72.98	15.46	15.35	11.85	12.50	6.44	9.48	4.44	3.66	20.79	3.92	52
76.50	14.23	14.48	12.88	11.76	8.27	7.47	5.22	5.00	20.68	0.60	67.7

**Table 10:** Applying CSO results to evaluate the deep learning algorithms (first dataset).

Algorithm	AUC	CAR	*F1*-score	Precision	Recall	FPR	PPV	NPV	MSE	Final result
*The results of the first dataset*										
ResNet50	1317.77	1404.60	1017.64	936.64	824.20	711.77	537.50	390.20	0.82	5715.99
DarkNet	1174.64	1307.39	957.15	869.42	742.66	643.42	498.72	354.63	1.45	5259.72
GoogleNet	1262.75	1387.56	1005.62	941.65	835.05	696.11	538.99	390.16	0.93	5664.74
MobileNetV2	1240.69	1357.00	986.16	869.84	805.39	643.03	507.89	376.23	0.80	5499.36
Xception	1090.73	1184.53	843.67	803.34	693.35	605.69	443.13	315.73	1.98	4766.83
VGG19	1165.93	1295.87	947.92	808.25	867.02	643.03	498.30	353.94	1.71	5292.50
VGG16	1181.02	1230.76	902.49	824.32	736.35	612.11	476.80	332.82	1.64	5070.82
InceptionV3	920.32	1013.29	728.85	693.84	601.52	493.12	387.91	275.79	1.16	4127.24
ResNet34	1314.28	1393.09	905.08	827.56	742.28	702.92	537.44	389.21	0.88	5405.14
CNNs	1269.72	1353.77	937.46	913.89	814.47	676.07	524.22	375.14	1.20	5511.41
DNN	1210.49	1310.92	914.30	872.34	793.81	657.28	501.28	357.62	1.33	5302.16
SAE	1166.94	1261.47	898.78	885.91	759.24	633.87	500.09	359.70	1.24	5197.02
InceptionResNetV2	1243.59	1350.70	968.39	914.83	780.65	674.35	525.41	369.43	2.06	5476.59
LSTM	1281.04	1390.47	993.69	931.63	824.48	680.38	536.85	379.38	2.02	5655.16
NASNet-Large	1151.99	1230.30	888.21	813.26	724.31	593.95	473.46	359.00	1.66	5044.91

*The results of the second dataset*										
ResNet50	1293.48	1290.40	1124.24	1041.93	725.85	664.05	463.27	451.61	1.12	5725.61
DarkNet	1170.09	1219.87	1075.52	967.16	681.18	628.43	434.35	412.17	1.55	5330.35
GoogleNet	1206.24	1256.51	1094.34	1001.61	704.01	640.08	434.98	421.77	1.22	5478.14
MobileNetV2	1182.90	1235.80	1085.06	991.85	690.69	633.73	444.22	416.07	0.97	5411.87
Xception	1207.23	1178.16	1032.60	940.36	665.37	603.64	419.26	404.87	1.26	5242.96
VGG19	1198.55	1230.58	1092.53	969.39	685.48	622.23	435.71	406.12	0.95	5395.18
VGG16	1299.88	1302.85	1143.83	1036.29	735.86	664.35	465.30	439.91	0.79	5758.79
InceptionV3	1027.64	1091.12	951.28	863.71	610.77	559.06	377.61	374.17	1.43	4735.81
ResNet34	1286.79	1277.51	1114.57	975.39	721.55	653.60	456.17	381.32	0.99	5558.71
CNNs	1213.79	1211.47	1071.01	970.45	676.38	615.29	432.05	413.67	1.03	5372.49
DNN	1166.39	1209.30	1061.60	977.15	679.36	620.67	427.72	414.17	1.72	5313.30
SAE	1182.62	1200.61	1055.16	945.53	672.32	611.11	424.69	406.87	1.61	5275.07
InceptionResNetV2	1257.76	1279.54	1126.81	1019.94	714.93	653.60	459.61	437.26	1.43	5640.84
LSTM	1173.23	1205.53	1061.08	970.80	687.38	618.05	430.90	396.17	2.05	5305.00
NASNet-Large	1154.30	1192.64	1037.24	942.94	667.44	607.15	426.36	410.77	1.28	5223.26

## Data Availability

Data derived from public domain resources are in references [19, 38].
